The article "Research on the Correlation between Multisource Big Data Virtual Assisted Preschool Education and the Development of Children's Innovative Ability" was published in 2022. Journal: Occup Ther Int.

# Research on the Correlation between Multisource Big Data Virtual Assisted Preschool Education and the Development of Children's Innovative Ability

**DOI:** 10.1155/2022/3880201

**Published:** 2022-04-27

**Authors:** Tuo Meimei, Long Baoxin

**Affiliations:** ^1^School of Education, Shannxi Fashion Engineering University, Xi'an, Shaanxi 712000, China; ^2^Shool of Education, Shannxi Normal University, Xi'an, Shaanxi 710062, China

## Abstract

**Objective:**

Innovation ability is an important part of children's core literacy and the core goal of science curriculum. As one of the important contents of scientific literacy, innovation ability is the key ability of young children to make informed decisions when facing scientific problems in social and personal life. In order to adapt to the future life, it is very important for children to have the ability to innovate. This research will provide a reference for the cultivation of children's innovative ability.

**Method:**

In the process of database design, certain design principles need to be followed. In this paper, the system and user experience are greatly optimized by reasonably constructing table structure, allocating storage space, and establishing indexes. In this system, the MySQL database is used to store system data, such as user registration information, subscription information, and system-provided services, and the data uploaded by users that needs to be processed is stored in Hive. Although the GFP algorithm can solve the problem of load balancing, when the largest conditional pattern base of a frequent item is projected to other nodes, a large amount of data transmission will occur, resulting in increased communication between nodes. In order to solve this problem, the FP-growth parallel algorithm based on traffic optimization gives priority to assigning each frequent item to the node that needs the least traffic when grouping it. *Results/Discussion.* Experiments show that the TFP algorithm not only satisfies the load balance of nodes but also ensures a small amount of communication between nodes, which is more efficient than the traditional FP-growth parallel algorithm. The survey results of the influencing factors of children's innovation ability match the theoretical hypothesis, and different influencing factors have different effects on each dimension of children's innovation ability. Through the basic fit index of the model, the evaluation of the external quality of the model and the test of the internal quality of the model, it is shown that the survey results of the influencing factors of children's innovation ability match the theoretical hypothesis. The three influencing factors of family participation and investment, teacher teaching, and peer collaboration and communication have a positive role in promoting children's innovation ability.

## 1. Introduction

With the gradual improvement of the construction of the kindergarten information system, more dimensions of education data are stored in the kindergarten database [1]. But for a long time, these data have not been valued by kindergartens. Their value is only to realize the simple query and statistical functions of the information system, and as the data is iteratively updated in the database, the new data gradually covers the old data. In the process, the value behind the data is also wasted as old data is erased [2].

In recent years, the popularization of the concept of big data and the development of data mining technology have made major kindergartens gradually realize the value behind educational data [3]. Through the analysis and mining of educational data, it helps school administrators to provide humanized and targeted guidance to children. Helping school leaders to formulate reasonable teaching policies and improve school management and teaching quality has become an important part of kindergarten construction [4].

The association mode reflects the knowledge of dependencies or associations between a transaction and other transactions. The most fundamental purpose is to find the association and derivation between data sets, in other words, to explore the association between items in a transaction. If there is a specific correlation between two or more items, then the known item value can be used to predict other unknown item values [5]. The core of association rule mining mainly includes two parts, the first is to find all frequent itemsets through continuous iteration, and the second is to obtain confidence and support from the obtained frequent itemsets and the support is not lower than the minimum confidence and minimum support [6].

Among the mining algorithms of association analysis, the Apriori algorithm is the most widely used association analysis mining algorithm and has great influence in identifying and mining frequent itemsets [7]. The Apriori algorithm was first used to solve the problem of association analysis. The algorithm mainly obtains the k+1 order frequent itemsets according to the frequent k itemsets. The database must be scanned every time until there is no frequent itemsets of the highest order [8]. The algorithm can study the association rules very efficiently, but when the support is small, the algorithm will have very significant defects, requiring multiple scans of the target database and a large number of useless candidate itemsets, which is too demanding on the performance of the system [9].

Through the research of big data, we can understand what children really lack and need and their preferred learning methods, and through technical analysis, we can find out what kind of courses are most attractive to children, and what kind of teaching mode can make them most happy to accept and learn. For teachers, they can also reduce work pressure and improve work efficiency through the teaching content provided by big data analysis [10]. For the principals, they can easily manage teachers and parents through big data technology. For parents, big data can allow them to understand their children's day-to-day learning, health, and teaching progress in the kindergarten, so as to achieve a better home coeducation. These are the models to be discussed in preschool education under big data [11].

The emergence of big data technology makes it possible to pay attention to the various performances of each preschooler—what children like to do, how long to do it, and what issues to discuss with classmates [12–14]. These data are mainly obtained through the observation of their class, homework, teacher-child interaction, and child-child interaction. These data are collected in a natural process. Observing the collected data will be more scientific and accurate in data analysis of children's various abilities, and of course, these theories will be more perfect and scientific [15]. This paper explores the external factors that affect young children's scientific reasoning, which will provide reference for the revision of children's scientific reasoning learning content standards, the evaluation and teaching improvement of innovation ability, and the construction of science education system inside and outside the school, so as to promote the development of children's innovation ability.

## 2. Methods

### 2.1. Hadoop Platform

Hadoop is an open source distributed system. Because Hadoop provides rich interfaces, developers can develop distributed applications without knowing too many low-level details and can use the interfaces to develop Hadoop-based data mining systems. Therefore, the Hadoop platform is currently the most commonly used implementation platform for parallel algorithms.

It includes multiple submodules, in addition to MapReduce, HDFS, but also Pig, Hive, etc. The structural framework of Hadoop is shown in Figure 1.

MapReduce is a parallel computing model that is often used to process large-scale data sets. It utilizes a cluster of multiple computers to simultaneously process parallelizable problems. MapReduce consists of two stages, Map and Reduce. The Map phase is responsible for data mapping, also known as data transformation. The Reduce stage is responsible for data aggregation. The execution process of MapReduce has the following six steps:

(1) We copied the MapReduce program to be executed to the master node Master and the child node Worker. (2) The master node Master decides the child nodes to execute the Map function and the Reduce function. (3) We allocate files on HDFS, project or divide the data set to each subnode and run the Map task in the subnode Worker. (4) We store the result of the Map function execution in the local disk where the child node is located. (5) The child node reads the Map result, adjusts and sorts the result, and executes the Reduce function. (6) The final result is output and written back to HDFS

### 2.2. System Database Design

The data stored in MySQL is mainly data related to user information, such as user information. At the same time, it also stores relevant data generated by user behavior, such as data cleaning records, data quality audit results records, user-defined quality audit standards, and other data.

The user id is stored in the user database table as the unique identifier of the user. The user name, password, email, etc. are all user registration information. The user balance will be deducted from the corresponding value when the user subscribes to the service, allowing a certain range of negative values. Users can read the list of all services provided by the system. The service list database table includes the service id as the unique primary key, as well as the service name, service price, and service introduction. After the user subscribes to the service, the subscription service will be stored in a subscription service database table, which uses the service id as the primary key and also includes the expiration time of the service and the value of the service access permission. The subaccount includes the account's parent account ID, login name, password, and account permission value.

For example, Table 1 is the data cleaning task table, which records the data cleaning tasks created by the user. Each cleaning task has a task task_id as a unique identifier. After the task starts, the start time and task status will be recorded. The data source cleaned by the user is recorded in the database, and the end time is written after the task ends.

Table 2 is the quality report form, which is the score record generated by the user after the quality assessment. The task_id is used as a unique identifier in the table. The report records the value of each indicator after the quality audit and evaluation and the score of each item, and the user can view it through the page.

Table 3 shows the data integration task table, which is a table that records the content of user integration tasks. The task_id is used as the unique identifier of the task, similar to the data cleaning table, and the fields include the number of workflow nodes, creator, creation time and end time, etc.

### 2.3. Parallelization Method Based on FP-Growth

When dealing with large-scale data sets, the disadvantage of the FP-growth algorithm is that it cannot build a memory-based global FP-tree, and the algorithm is time-consuming to recursively mine conditional FP-trees. In order to solve the limitations of the algorithm in time and space, the idea of “data decomposition” is usually used to design a parallel FP-growth algorithm [16].

The basic idea of data decomposition is to divide and conquer. For any original data set *D*, when the size of *D* is smaller than the available memory capacity *M*, a certain memory-based association rule algorithm generate association is used to mine association rules, such as FP-growth. When the size of *D* exceeds the memory, a certain decomposition strategy is used to decompose *D* into k subdata sets *D*1, *D*2, ⋯, *Dk*, and then, the data decomposition algorithm is recursively called for each *Dk*. Since the mining results of each subdata set are part of the full-set data mining results, the combine function combines the results of each subdata set to obtain the mining results of data set *D*. The decomposition strategy divides the large-scale data set into small-scale data subsets. Such a division can solve the time and space limitations of the FP-growth algorithm, which are mainly reflected in the following two aspects:

1. The FP-tree of each subdata set will be much smaller than the global FP-tree of the original data set. Therefore, it can be put into the memory of each processing node for calculation, which effectively solves the problem that the global FP-tree cannot be read into the memory at one time when the data set is too large
2. The time complexity of recursively mining conditional FP-trees in the classical FP-growth algorithm is high, but the subdata set can mine its local conditional FP-trees in parallel on each processing node, which can reduce the execution time of the algorithm

The process of counting frequent 1-itemsets is similar to counting statistics, so the partitioning strategy in data decomposition can be used for data set decomposition. Each processing node needs to count the frequency of the data items divided into the local data set to obtain the local itemset count. Then, each node communicates with each other to obtain the global frequency of each item and deletes the nonfrequent itemsets according to the minimum support threshold to obtain the frequent 1-itemsets. Broadcast the frequent 1-itemsets to each child node to ensure that each child node saves a list of frequent 1-itemsets [17–19].

After getting the list of frequent 1-itemsets, it is necessary to build a global FP-tree to obtain the conditional pattern basis of each item. When the data set is too large, the global FP-tree cannot fit into the memory [20, 21]. Therefore, the parallelized method decomposes the data set into subsets, builds FP-tree on the data subset, which is called “local FP-tree”, and then calls the FP-growth method for the local FP-tree to recursively mine the local association rules.

When constructing a local FP-tree, the association information between itemsets is not damaged. For any item, its conditional pattern base is certain. The algorithm does not need to generate a global FP-tree, but only needs to send the conditional pattern base of each item to the specified computing node, and then build the conditional FP-tree of the item on the node, and use the FP-tree for association rule mining. When the data set and the minimum support threshold are fixed, multiple local FP-trees can also mine the same association rules as the global FP-trees.

### 2.4. Design of TFP Association Algorithm Based on MapReduce

For each piece of sample data, we can use “1 frequent itemset” to find out the frequent items, and the generated GF-List table can project each item into a certain group, denoted as gid. For each 1 frequent term, find all conditional pattern bases with it as a suffix pattern. The data is distributed according to the gid corresponding to the item, that is, the gid is used as the key, and all conditional pattern bases are used as the value. The items of the same gid and its conditional pattern base set will be concentrated in a reducer task. In the reduce function, a local conditional pattern tree is established for the conditional pattern base, and the FP-growth algorithm is recursively called to obtain frequent itemsets. The traditional FP-growth algorithm is the same.

FreqItemCountJob is used to generate 1 frequent itemsets. That is, the frequency of each item is counted, and elements less than the minimum support degree are deleted. The Mapper class is used to split the data to get an array of items and convert the array into an output format where the item is the key and the value is 1. The Reducer class is used to collect the value of the same item and accumulate the sum to get the frequency of the item. If the frequency is greater than the minimum support degree, the result will be output; otherwise, it will not be output.

SortJob sorts the above output results, that is, arranges the set of 1 frequent items in descending order of frequency from large to small. Because the Reducer has its own mechanism for sorting according to the Key value when outputting, we use this mechanism to achieve sorting. But because Reducer excludes Key values, we need to swap the positions of Key and Value in Mapper. The InverseMapper.class class is a class library provided by Hadoop to swap Key and Value. SortJob does not require additional processing by the Reducer class, so just set sortJob.setNumReduceTasks(1).

FPgrowthJob is used to mine association rules in parallel. This is the second scan of the database. For each transaction, the Mapper class will extract all the conditional schema bases of each item in turn and output them in the format with gid as Key and conditional schema base as Value. In addition, Hadoop provides a mechanism for global variables, namely, DistributedCach, using which all Mappers or Reducers can share global variables. Because the <item-gid> projection table will not be very large, we use DistributedCache in the setup function of the Mapper class to read the projection table. The Reducer class aggregates the conditional pattern bases of the same group of items to build a local conditional pattern tree (local FP-tree), and uses traditional FP-growth to perform rule mining on the tree, and outputs the rule pattern and the support of the rule. The pseudocode of the Reduce function in the association rule mining process is shown in Table 4.

### 2.5. Selection of Research Samples

Due to the influence of objective factors, this paper adopts a nonrandom sampling method. In order to ensure that the sample is as comprehensive as possible, we have visited 6 public kindergartens, involving a total of 5 regions. According to the grades of kindergartens, the samples include provincial demonstration gardens, municipal demonstration gardens, and national high-quality gardens. The age distribution of the survey samples is shown in Figure 2.

### 2.6. Checking Method of Children's Daily Activities

The theory of multiple intelligences advocates that the human intelligence structure is composed of at least nine kinds of intelligence elements, and each person has nine relatively independent intelligences at the same time, and the combination of different ways and different degrees makes each person's intelligence unique, forming an interindividual intelligence.

Cognitive development in early childhood is mainly the development of children's thinking ability. The thinking of young children is different from that of adults. Through Piaget's theory of cognitive development stages, we know that children under the age of 7 mostly adopt concrete conceptual thinking but have not yet developed the abstract thinking of older children and adults. Children use innate physical and mental tools to understand the world through interaction with the surrounding environment, and in the process of interaction, they construct the concept of the world.

When children manipulate objects in their environment, they learn to respond differently to different objects. The new knowledge acquired is also integrated into the existing knowledge, which contributes to the development of their way of thinking. Children's cognitive development stems from physical maturity, from their interaction with the environment and their spontaneous discovery of the environment.

The main aspects of child development are often defined as emotional, social, physical, cognitive, and linguistic, often ignoring the development of creativity. Every child has the potential to become an artist, musician, writer, or inventor, and their interests will lead them in the direction of their own if the teacher does not hinder or inhibit their behavior.

The creativity of young children is understandable because what they say and do is new to them, and they explore, experiment, merge, separate, and manipulate objects in ways that adults never thought possible. They use imagination as a tool to create fantasy situations or the ability to realize fantasies by pretending or imagining the role of others. Early childhood specialists have come to recognize that imagination is one of the most effective means of promoting a child's intellectual, social, language, and especially creative development. Their creativity is often reflected in artistic activities and social performance game activities.

### 2.7. Interview Outline Design

According to the interviewees, this paper designs an interview outline for young children and an interview outline for kindergarten teachers (including the principal and other managers). The purpose of the interview is mainly to investigate the content that is not easy to observe, such as the emotional experience behind the behavior, so as to ensure a comprehensive study of the survey questions.

The interviews with young children mainly include inquiries in terms of participation in activities, social interaction and emotional experience, attachment relationship with primary caregivers and teachers, and self-concept formed. In addition, a general understanding of the activities they participate in outside of kindergarten is required. Although there are still doubts about the subjectivity of the interview method, the author believes that what we often seek is not the absolute truth, but the “truth” in the eyes of the respondents.

For teachers and kindergarten managers, interviews can be more in-depth than children. The main purpose is to have a more objective understanding of the innovative development of young children from the perspective of teachers and other staff. This is a major part, and it is necessary to see through the eyes of educators whether young children are innovative, what aspects of their innovation are manifested in, and where the “proximal development zone” of their innovative quality development is. Through a series of questions, we can not only know how well educators understand children's innovative quality but also explore teachers' own educational concepts and educational experience. In addition, it is also necessary to know what efforts the kindergarten has made for the development of children's innovative quality through interviews with teachers, and what shortcomings still exist.

## 3. Results

### 3.1. Cluster Environment

The cluster environment is built on the Hadoop platform, and the number of nodes is 5. The detailed parameters of the hardware and software environment used to test the algorithm are shown in Table 5. During the test, use ssh under the Xshell software to remotely log in to the server locally, upload the program jar package and input data to the server through the scp command, and upload the input data to HDFS using the dfs command.

### 3.2. Correlation Algorithm Simulation Results and Analysis

When the amount of data is small, the job scheduling time accounts for a larger proportion of the total running time. And, as the number of Reduces increases, the time of the two parallel algorithms decreases more and more slowly, and when the number of Reduces is greater than 10, the program running time remains almost unchanged. This is because when the number of Reduces increases, the communication overhead also increases. The variation of the running time of the PFP algorithm and the TFP algorithm with the number of reducers is shown in Figure 3. From the graph, we can see that the TFP algorithm performs slightly better than the PFP algorithm in terms of running time.

For the data set webdocs.dat, this paper sets the minimum support to 5%, and the number of groups for the TFP algorithm is 5 groups. In a stand-alone environment, the traditional FP-growth algorithm will cause memory overflow, so it cannot run. However, in a distributed environment, both the PFP algorithm and the TFP algorithm can run successfully, indicating that the parallel algorithm can indeed solve the problem of traditional FP-growth memory overflow. On large data sets, the running time of the TFP algorithm is significantly smaller than that of the PFP algorithm, indicating that the TFP algorithm is more efficient on large-scale data sets. Moreover, when the number of Reduces is greater than 20, the running time of the PFP algorithm increases, while the change of the TFP algorithm is relatively stable, indicating that the stability of the TFP algorithm is better.

In this paper, data sets of different sizes are used for experiments, and the number of Reduces is set to 10, the minimum support degree is 5%, and the number of groups of TFP algorithm is 5. The running times of the PFP and TFP algorithms are shown in Figure 4, respectively, with different data set sizes. It can be seen that the running time of the TFP algorithm is shorter than that of the PFP algorithm, and as the data set increases, there is a gap in the running time of the two. This shows that in the application of large-scale association rule mining, TFP algorithm has better applicability and scalability than PFP algorithm.

In this paper, when the data set is 2000 MB, the load of each Reduce task is tested, and the execution time of the Reduce node is used to represent the load in the experiment. The TFP algorithm can better realize the load optimization of nodes, thereby improving the overall execution time.  Figure 5 shows the correlation between the size of the multisource data set and the development of children's innovative ability.

### 3.3. Evaluation of the Development of Children's Innovative Ability

The fitness indicators of the model are sorted and listed in detail in Table 6. It can be seen from the table that the chi-square value of the overall fitness of the model for influencing factors of children's innovation ability is equal to 212.341 (*P* = 0.0001 < 0.05), which does not meet the overall model fitness test. When judging the fitness of the overall model, since the chi-square value is easily affected by the sample size, the larger the sample observation value is, the larger the model chi-square value will be. The conclusion of rejecting the null hypothesis is formed. Therefore, if the number of samples is large, other fitness statistics should be referred to in the judgment of the overall model fitness, not only the chi-square value. In this study, the number of samples participating in the survey is relatively large, so the chi-square value is only used as a reference, not as an indicator of whether the test is passed.

From other fitness indicators, the ratio of chi-square degrees of freedom is 2.991<3.000, the standard square root residual RMSEA = 0.041 < 0.05, the fitting index GFI value = 0.974 > 0.90, the adjusted fitting index AGFI value = 0.962 > 0.90. These indicators all reach the acceptable standard of the model. Taking into account other fitness indicators, from the perspective of absolute fitness level, value-added fitness level, and parsimonious fitness level, the theoretical causal model diagram of the influencing factors of children's innovation ability can be adapted to the actual data.

## 4. Discussion

### 4.1. Analysis of the Preschool Education Curriculum Itself

The suitability of the curriculum itself and the richness of curriculum resources can affect the effect and quality of curriculum implementation [22]. Innovative preschool education curriculum that conforms to the characteristics of children's physical and mental development can help children achieve better development.

The innovative curriculum of preschool education is mainly based on the text teaching materials provided. The clarity and feasibility of the content of the teaching materials affect the way and effect of teachers' curriculum implementation [23–25]. To introduce change into educational practice, the success or failure of the introduction process is closely related to the state of the new curriculum plan itself. Specifically, if the newly compiled kindergarten curriculum itself is of high quality, disseminated, operable, and in line with actual needs and public awareness, then the effectiveness of curriculum implementation will increase. The innovative curriculum of preschool education has strong integration, and the design and implementation of the curriculum have certain complexity and difficulty. Through observation, it is found that kindergartens lack kindergarten-based preschool education innovative courses, and the existing teaching materials for implementing courses do not clearly mention clear activity goals and specific implementation methods [26, 27]. The existing preschool teachers' ability and material support are difficult to achieve, and the unreasonable and inappropriate curriculum text will hinder the implementation of the curriculum. Curriculum resources are the basis and important guarantee for curriculum implementation. The abundance of curriculum resources is an important factor affecting curriculum implementation. Rich curriculum resources can promote and positively influence children's learning.

Through observation, it is found that the kindergarten provides a variety of resource support for children's innovative preschool education curriculum learning, such as cardboard boxes, paper cups, scientific experimental equipment, and other materials, which can basically guarantee the implementation of the existing curriculum. However, there are still many existing curriculum resources that need to be excavated and enriched, and the lack of tools and materials in engineering and technology inhibits the learning of relevant knowledge and experience for young children.

### 4.2. Analysis of Teachers' Factors in the Development of Innovation Ability

Kindergarten teachers are the implementers of innovative courses in preschool education, and they are the key factors affecting the implementation of courses. The main factors of curriculum implementation are teachers' motivation, teachers' autonomy, teachers' sense of commitment, teachers' beliefs, teachers' sense of security, teachers' time, teachers' abilities, teachers' culture, teachers' practical knowledge, and so on. In addition to providing a rich learning environment and resources, teachers' knowledge, effectiveness, and attitudes toward science are also identified as important factors affecting early childhood STEM education. In terms of teacher factors, it mainly analyzes from four aspects: teacher's belief, teacher's attitude, teacher's knowledge, and teacher's ability.

Based on the perspective of teacher development, teachers' belief is the spiritual pillar of teachers' life, the creed of teachers' profession, the core elements of teacher culture, the hidden guide of teachers' behavior, and the inner driving force of teachers' development. Teachers' beliefs about STEM (science, technology, and math) and its appropriateness in early childhood influence their decisions and behaviors, including the time and attention devoted to learning STEM in the classroom [28–30]. Teachers' beliefs guide teachers' behavior, and firm teacher beliefs are the driving force for the implementation of innovative preschool education courses.

Teachers' cognition and attitude towards curriculum can affect the quality of curriculum implementation. Different teachers have different attitudes towards implementing innovative preschool education curriculum, resulting in differences in curriculum implementation behavior [31]. Through interviews and observations, it was found that teachers' behaviors were mainly divided into two types: one was ignoring the inquiry process, and the other was exploring together with children.

The media and science and technology interest classes that parents and young children communicate about science-related content, conduct scientific practice, and invest in acquiring scientific and technological information will have a positive role in promoting the development of young children's innovative ability. Science teachers' use of inquiry-based teaching, teaching of scientific reasoning content (methods), and metacognitive teaching of scientific reasoning, and teaching of the nature of science will positively promote the development of children's innovative ability. The exchange of scientific content and scientific practice with peers in and out of class will positively promote the development of children's innovative ability.

A teacher's knowledge and skills are one of the most important factors in determining how much content a child can learn, and it has a significant impact on a child's learning and development. Teachers' knowledge is transformed into knowledge learned by children through the implementation of specific activities, so the structure and richness of professional knowledge of preschool teachers are very important. In the “Professional Standards for Kindergarten Teachers,” promulgated by the Ministry of Education, the professional knowledge of kindergarten teachers is divided into three parts: “Knowledge of Early Childhood Development,” “Knowledge of Early Childhood Care Education,” and “General Knowledge.” Teachers can only support early childhood development if they have sufficient and broad knowledge. The implementation of innovative curriculum in preschool education relies on teachers' knowledge base of science, technology, engineering, and mathematics, but in practice, preschool teachers' knowledge of science, technology, engineering, and mathematics is relatively weak [32, 33].

The ability of kindergarten teachers plays a vital role in kindergarten education activities, and kindergarten teachers must have the ability to plan and implement courses. Transforming specific activity plans into practical educational activities requires teachers to observe and guide children's behavior during activities, provide children with opportunities for exploration and cooperation, and promote children's active learning. In the process of implementation, teachers' language expression ability, activity organization ability, and so on are fully tested. Through observation and interviews, it is found that there are differences in curriculum implementation ability of preschool teachers in different areas of focus and teaching age.

### 4.3. Analysis of Child Factors

Differences in the existing experience of different children will also affect the learning effect of children in the implementation of the curriculum [34, 35]. Some children are more interested in scientific activities and actively learn relevant knowledge in daily life and at home. An observed child in a large class likes to visit science and technology venues in his spare time, has a high interest in science learning, and performs well in kindergarten. Therefore, children with different knowledge and experience have different acceptance and learning enthusiasm for STEM curriculum activities, which can affect the effect of innovative curriculum implementation in preschool education [36].

According to the existing kindergarten class setting, from the perspective of teacher-to-child ratio, each class in the existing class is equipped with three full-time teachers, and the number of children in the class is about 40. In the implementation process, one teacher is the main organizer, and the other two teachers serve as teaching assistants. However, due to the current situation of the number of children, there are difficulties in group work and activity organization order.

### 4.4. Kindergarten Factors

Kindergarten is the field for the implementation of innovative courses in preschool education. In addition to basic space, materials, and teacher support, its smooth implementation depends on the effective organization and top-level arrangements of kindergarten managers [37]. For example, kindergarten curriculum leaders and kindergarten teaching research and training will implement the curriculum.

Curriculum leadership of the kindergarten principal is the ability of planning, execution, construction, and evaluation that is reflected in the course practice process in order to improve the quality of the kindergarten curriculum by the curriculum team with the principal as the core. The state of the principal's curriculum leadership determines and affects the overall implementation of curriculum leadership in kindergartens. The curriculum leadership of the kindergarten principal includes the ability to interpret the kindergarten curriculum, the ability to judge the current situation of the kindergarten curriculum, the ability to develop curriculum resources, the ability to plan the implementation of the curriculum, and the ability to construct the curriculum culture.

In order to become a real curriculum decision-maker, the principal of the kindergarten should grasp the characteristics of the kindergarten to conduct curriculum leadership, promote strengths but not avoid weaknesses, and realize the in-depth combination of theory and practice. Based on the development needs of the kindergarten and the actual situation of the existing kindergarten curriculum, the organization and arrangement of the STEM curriculum implementation by the kindergarten director reflects his strong curriculum leadership.

In terms of the kindergarten's understanding of the innovative curriculum of preschool education, the principal agrees with project learning, the main implementation method of the innovative curriculum of preschool education, and believes that it can bring a new way of learning to children. In the process of implementing the innovative curriculum of preschool education, the old teachers have the characteristics of “strong ability and old ideas,” and the young teachers have the characteristics of “weak ability and new ideas.” It is difficult for the old teachers to change their ideas, and the difficulty for young teachers is the lack of professional ability.

Therefore, the implementation of innovative preschool education courses has different values and roles for elderly teachers and young teachers. The fundamental starting point is to promote the transformation of old teachers' ideas and the improvement of young teachers' abilities, and to strengthen the construction of teachers in kindergartens. Kindergarten's reasonable positioning and implementation arrangements for innovative preschool education courses, as well as the overall allocation of teacher resources and curriculum resources, have a positive impact on curriculum implementation.

Kindergarten teaching and research activities are an efficient way for teachers to improve teachers' professional knowledge and implementation ability in a short period of time. Regular high-quality teaching and research activities play a role in promoting the quality of curriculum implementation and teachers' professional development [38]. The theme, content, practice and frequency of teaching and research activities, and participants in teaching and research activities will affect the effect of teaching and research, thereby affecting teachers' understanding of innovative preschool education curriculum and behavior improvement.

In terms of teaching and research, in the teaching and research activities of kindergartens, the group summarizes and reflects on the course implementation process, and teachers collectively learn and reflect on the difficulties and experiences in the implementation of innovative courses in preschool education and present and report in the form of course stories [39, 40]. In the two teaching and research activities on the innovative curriculum of kindergarten preschool education that the researchers participated in, they mainly analyzed and discussed teachers' curriculum stories during the course implementation process, and there were few teaching and research activities on the curriculum content itself and teachers' professional knowledge and ability.

## 5. Conclusion

Although the GFP algorithm can solve the problem of load balancing, when the largest conditional pattern base of a frequent item is projected to other nodes, a large amount of data transmission will occur, resulting in increased communication between nodes. To solve this problem, the TFP algorithm prioritizes the nodes that require the least amount of traffic when grouping each frequent item. Experiments show that the TFP algorithm not only satisfies the load balance of nodes but also ensures a small amount of communication between nodes, which is more efficient than the traditional FP-growth parallel algorithm. At the end of the paper, the TFP algorithm is compared with the traditional no-load optimized PFP algorithm. The experiments show that the TFP algorithm is superior to the PFP algorithm in terms of time efficiency, adaptability, and scalability, especially when the data scale becomes larger, and the TFP algorithm can show a greater advantage. The three potential external factors have different main promoting effects on innovation ability. The media of family participation and investment in obtaining scientific information and the investment interest class have a relatively large role in promoting the innovation ability in the dimension of “asking questions,” and teacher teaching has a relatively large role in promoting the innovation ability in the dimension of “reasoning and drawing conclusions.” In addition, except for the dimension of “asking questions,” the influence of peer collaboration and communication on the ability of the other three dimensions of innovation ability is relatively larger than the other two factors.

## Figures and Tables

**Figure 1:** Hadoop structural framework.

**Figure 2:** The age distribution of the survey samples.

**Figure 3:** Comparison of algorithm running time under different numbers of Reduces based on the data set accidents.dat.

**Figure 4:** Comparison of algorithm running time with different data set sizes.

**Figure 5:** Correlation between the size of multisource data sets and the development of children's innovative ability.

**Table 1:** Data cleaning task table.

Field name	Type	Primary key	Empty	Field description
Description	varchar(512)	N	N	Mission details
end_time	varchar(256)	N	Y	End time
Status	varchar(1024)	N	N	Task status
Creator	varchar(64)	Y	N	Task creator
datasource_id	int	N	N	Data source id
task_id	varchar(64)	N	N	As a unique identifier for the task
create_time	int	N	Y	Creation time

**Table 2:** Quality report form.

Field name	Type	Primary key	Empty	Field description
Score	Float	N	N	Overall rating
Timeliness	varchar(1024)	N	N	Timeliness score
Consistence	Float	N	N	Consistency score
Accuracy	Float	N	N	Accuracy score
Effectiveness	int	N	N	Effectiveness score
Completeness	varchar(64)	N	N	Integrity score
Uniqueness	Float	N	N	Uniqueness score

**Table 3:** Data integration task table.

Field name	Type	Primary key	Empty	Field description
task_id	Float	N	N	id
create_time	varchar(256)	N	N	Creation time
last_modify_time	Timestamp	N	N	Last modified
args	Float	N	N	Rule parameters
Enabled	int	N	N	Whether to enable
end_time	Timestamp	N	N	End time
running_wf_num	varchar(512)	Y	N	Number of running workflow nodes

**Table 4:** Pseudocode of Reduce function in association rule mining process.

Step	FPgrowthReducer.class public void map (LongWritable key, Text value, Context context){
1	Split each row of value by, and store them in the arr array;
2	Create a new LinkedList collection list;
3	Use the for loop to read out the arr array sequentially {
4	If an item ele in the arr array is in the frequent 1 itemset; {
5	Write the ele to the list collection;
6	New LinkedList<List<String>>linked list trans;
7	Create a new String array arr;
8	Assign the array to values divided by \t;
9	Declare and initialize a new LinkedList<String> linked list list;
10	Use the for loop to read out the contents of the arr array in turn;
11	Add each item ele to list;
12	Add list to collection trans; }}

**Table 5:** Distributed cluster environment.

Systems and applications	Illustrate
Apache	Apache-tomcat-6.0.37
Hadoop	Hadoop 2.3.1
Linux	Centos 6 (x86_64)
JDK	JDK-6u37-linux-i586
192.168.3.156	DataNode, TaskTracker
192.168.3.157	Cores(CPU): 8 cores
192.168.3.158	RAM: 32GB
192.168.3.159	Hard disk size: 2400GB
192.168.3.160	

**Table 6:** The overall model fit index of the structural model analysis of the influencing factors of children's innovation ability.

Statistical test	Fitting criteria or thresholds	Test result data	Model fit judgment
PGFI	>0.50	0.76	Y
PNFI	>0.50	0.79	Y
PCFI	>0.50	0.82	Y
CN	>220	550	Y
GFI	>0.9	0.97	Y
AGFI	>0.9	0.98	Y
NFI	>0.85	0.92	Y
RFI	>0.85	0.91	Y
IFI	>0.85	0.94	Y
TLI	>0.85	0.98	Y

## Data Availability

The data used to support the findings of this study are available from the corresponding author upon request.
